# Different Effects of Hematoma Expansion on Short-Term Functional Outcome in Basal Ganglia and Thalamic Hemorrhages

**DOI:** 10.1155/2021/9233559

**Published:** 2021-10-25

**Authors:** Lijing Deng, Kai Chen, Liu Yang, Zhaoxu Deng, Haijun Zheng

**Affiliations:** ^1^Department of Neonatology, Shenzhen Third People's Hospital, Second Hospital Affiliated to Southern University of Science and Technology, Shenzhen, Guangdong Province, China; ^2^Department of Medical Imaging, Shenzhen Samii Medical Center, Shenzhen, Guangdong Province, China; ^3^Department of Neurology, The First Affiliated Hospital of Jinan University, Guangzhou, Guangdong Province, China; ^4^Department of Radiology, The Second Affiliated Hospital of Xiangnan University, Chenzhou, Hunan Province, China; ^5^Department of Radiology, Suxian Hospital Affiliated to Xiangnan University, Chenzhou, Hunan Province, China

## Abstract

**Purpose:**

To investigate the impact of hematoma expansion (HE) on short-term functional outcome of patients with thalamic and basal ganglia intracerebral hemorrhage.

**Methods:**

Data of 420 patients with deep intracerebral hemorrhage (ICH) that received a baseline CT scan within 6 hours from symptom onset and a follow-up CT scan within 72 hours were retrospectively analyzed. The poor functional outcome was defined as modified Rankin score (mRS) > 3 at 30 days. Receiver operating characteristic (ROC) curves for relative and absolute growth of HE were generated and compared. Multivariable logistic regression models were used to analyze the impact of HE on the functional outcome in basal ganglia and thalamic hemorrhages. The predictive values for different thresholds of HE were calculated, and correlation coefficient matrices were used to explore the correlation between the covariables.

**Results:**

Basal ganglia ICH showed a higher possibility of absolute hematoma growth than thalamic ICH. The area under the curve (AUC) for absolute and relative growth of thalamic hemorrhage was lower than that of basal ganglia hemorrhage (AUC 0.71 and 0.67, respectively) in discriminating short-term poor outcome with an AUC of 0.59 and 0.60, respectively. Each threshold of HE independently predicted poor outcome in basal ganglia ICH (*P* < 0.001), with HE > 3 ml and > 6 ml showing higher positive predictive values and accuracy compared to HE > 33%. In contrast, thalamic ICH had a smaller baseline volume (BV, 9.55 ± 6.85 ml) and was more likely to initially involve the posterior limb of internal capsule (PLIC) (85/153, 57.82%), and the risk of HE was lower without PLIC involvement (4.76%, *P* = 0.009). Therefore, in multivariate analysis, the effect of thalamic HE on poor prognosis was largely replaced by BV and the involvement of PLIC, and the adjusted odds ratios (ORs) of HE was not significant (*P* > 0.05).

**Conclusion:**

Though HE is a high-risk factor for short-term poor functional outcome, it is not an independent risk factor in thalamic ICH, and absolute growth is more predictive of poor outcome than relative growth for basal ganglia ICH.

## 1. Introduction

Spontaneous intracerebral hemorrhage (ICH) is a catastrophic form of stroke associated with high mortality and severe disability among survivors. The functional outcome after ICH depends on the hematoma volume and location [1]. Since hematoma expansion (HE) is common in acute ICH and correlates with early deterioration and poor functional outcome [2, 3], it is a promising prognostic/therapeutic index. However, most studies so far considered hematoma growth > 6 ml or >33% as the thresholds for defining HE [4–7]. This limits the predictive power of HE since a particular threshold may have different prognostic impacts depending on the ICH location. Localized and deep ICH usually has a worse clinical outcome [8], especially thalamic ICH and that involving posterior limb of internal capsule (PLIC) [9, 10]. In addition, the risk of HE is also associated with the hemorrhage location [11, 12]. Since lobar ICH with larger volume has specifically better outcomes [13, 14], it is necessary to further explore the impact of HE on the prognosis of deep ICH. Although thalamus and basal ganglia share a similar “deep” geographical location, their neuroanatomical functions are substantial different. Nakagawa et al. [15] found that thalamic hemorrhage has smaller hematoma volume thresholds than basal ganglia hemorrhage in predicting poor functional outcome. Also, there is currently no scientific consensus on the definition of HE [16]. Dowlatshahi et al. suggested that the absolute growth thresholds of HE have a predictive performance for severe outcomes compared to relative thresholds [17]. However, another study showed that absolute growth thresholds may have limited predictive power due to largely different baseline hematoma volumes [18]. Therefore, we hypothesized that the prognostic impact of hematoma growth thresholds differs in thalamic ICH and basal ganglia ICH, and it may provide important insights for assessing acute deep ICH.

## 2. Methods

### 2.1. Study Population

Data of patients with supratentorial ICH was collected from 4 hospitals (the First Affiliated Hospital of Jinan University, Affiliated Hospital of Xiangnan University, the Second Affiliated Hospital of Xiangnan University, and Su Xian Hospital Affiliated to Xiangnan University) from January 2015 to May 2019. The patients had received a baseline CT scan within 6 hours after symptom onset and a follow-up CT within 72 hours. Patients younger than 18 years and those with nonparenchymal hemorrhage, infratentorial and lobar location, secondary hemorrhage, and multiple hemorrhage were excluded. In addition, patients that underwent surgery for hematoma evacuation prior to the follow-up CT and with premorbid modified Rankin scale scores > 3 were also excluded (Figure 1). To better assess the prognostic impact of HE at different ICH locations, patients with preceding anticoagulant use or coagulopathy on admission were also excluded. The baseline data included age, gender, time from symptom onset to baseline CT, Glasgow Coma Scale (GCS) score, systolic and diastolic blood pressure (BP) on admission, current smoking, daily alcohol drinking, antiplatelet medications, history of diabetes, platelet count, international normalized ratio (INR), baseline hematoma volume, PLIC involvement, ICH location, presence of intraventricular hemorrhage (IVH) and HE, treatment method, and modified Rankin scores (mRS) at 30 days. The study was approved by the local ethics boards, and informed consent was not required due to the retrospective nature of the study.

### 2.2. Image Analysis/Definitions of HE

The 3D-Slicer platform (version 4.10.1, http://www.slicer.org) was used for image analysis and calculation of ICH volume. DICOM data of all CT scans were imported into 3D-Slicer, and the entire hematoma was free-hand segmented on consecutive axial CT slices by a radiologist. The total hematoma volume was calculated as the sum of all voxel sizes in the segmented regions. IVH was not included in calculating the hematoma volume. Signs of ICH in the baseline CT scans were analyzed by two radiologists in a blinded manner. The deep regions of ICH were divided into the thalamus and basal ganglia (since 3 sites caudate head, lentiform nucleus, and thalamus are well delimited in CT imaging, the site of basal ganglia just included the caudate head and lentiform nucleus). If the hemorrhage extended to the other deep region or lobar, the volume of hemorrhage at the origin should be more than three times greater than the other areas. Any bleeding extended to PLIC was defined as involvement and was analyzed as an independent factor in the logistic regression analysis.

Besides the most commonly used definitions of HE (absolute growth > 6 ml and relative growth > 33%), we generated receiver operating characteristic (ROC) curves for absolute and relative growth and compared them; the method of Youden [19] was used to select the optimal cutoff for growth. Then, a small threshold of HE for both thalamic ICH and basal ganglia ICH was determined by considering the optimal cutoff points of ROC curves and the minimal detectable difference (MDD) which was used to avoid errors of hematoma volume measurements [17].

### 2.3. Statistical Analysis

Normally distributed continuous variables were presented as mean ± standard deviation (SD), and skewed continuous variables as medians and interquartile ranges (IQR). Categorical variables were presented as percentages. Baseline characteristics were compared by the chi-square test, Fisher's exact test, Student t test, or Mann–Whitney *U* test as appropriate. *P* < 0.05 was considered statistically significant. Odds ratios (OR) and 95% confidence interval (95% CI) were calculated for each factor. The possible risk factors with *P* < 0.1 in the univariate analyses were included in the multivariate logistic regression model. The likelihood ratio test was used to assess the significance of the model. The same analysis was repeated after adjusting for each of the three HE thresholds. Finally, a correlation coefficient matrix was used to determine the relationship between the covariates in the logistic regression model. All statistical analyses were performed with R software (version 3.6.0, R Foundation for Statistical Computing, Vienna, Austria).

## 3. Results

A total of 420 patients met the inclusion criteria, of which 147 (35%) exhibited thalamic ICH and 273 had basal ganglia ICH (65%). Patients with basal ganglia ICH were younger (median: 59 years, *P* < 0.001) and exhibited larger hematomas, lower probability of PLIC involvement and presence of IVH in both the baseline and follow-up CT, and higher incidence of absolute growth (>6 ml) of HE (*P* ≤ 0.001) compared to the thalamic ICH group. Other baseline characteristics were similar for both anatomical locations (Table 1). After excluding 21 patients (13 were transferred to other hospitals and 8 withdrew treatment in critical condition), 399 patients (141 with thalamic ICH and 258 with basal ganglia ICH) were included in the subsequent analysis. Thirty-eight patients underwent external ventricular drainage (a higher proportion in the thalamic ICH group, 23/141 or 16.31%, *P* = 0.001), and 52 patients received a hematoma stereotactic evacuation or an additional craniectomy (a higher proportion in the basal ganglia ICH group, 46/258 or 17.83%, *P* < 0.001). Furthermore, 53.38% of the patients (213/399) exhibited mRS > 3 at 30 days, and the difference in proportion between the two groups was not significant (*P* = 0.067).

ROC curves for absolute and relative hematoma growth, for the prediction of mRS > 3, are shown in Figure 2. The area under the ROC curve (AUC) for absolute and relative growth was 0.59 and 0.60 in thalamic ICH, which was lower than that in basal ganglia ICH, where the AUC for absolute and relative growth was 0.71 and 0.67, respectively. HE discriminated the risk of poor outcome only modestly. Absolute growth was more predictive of poor outcome than relative growth (*P* = 0.001) in basal ganglia ICH, but there was no significance between the AUCs for absolute vs. relative HE in thalamic ICH. According to the method of Youden, the best cutoff for absolute growth was 0.88 ml (sensitivity 42.9%, specificity 82.5%) in thalamic ICH and 3.86 ml (sensitivity 55.8%, specificity 87.6%) in basal ganglia ICH. Considering the different cutoff points of both, we chose the threshold of 3 ml to redefine HE, which also could exceed the MDD.

The predictors of the poor functional outcome for thalamic and basal ganglia ICH are summarized in Tables 2 and 3 , respectively. As per the univariate analysis, HE was significantly associated with mRS > 3 regardless of the location. Furthermore, the patients with mRS > 3 at 30 days were older than those with mRS ≤ 3 (67 vs. 62 in thalamic ICH, *P* = 0.01; 60 vs. 55 in basal ganglia ICH, *P* < 0.001). A lower GCS score, a higher baseline ICH volume, PLIC involvement, and presence of IVH were also associated with increased risk of poor functional outcome.

Three HE thresholds were, respectively, analyzed in multivariable logistic regression models to assess the correlation of each with the poor functional outcome. Each threshold of HE was an independent predictive factor for the poor functional outcome of basal ganglia ICH (*P* < 0.001), whereas none independently impacted the prognosis of thalamic ICH (*P* > 0.05). All adjusted OR values are summarized in Tables 2 and 3. Other independent risk factors were age, GCS score, baseline ICH volume, and PLIC involvement, whereas IVH was an independent factor of mRS > 3 only in patients with basal ganglia ICH (OR 3.16, 95% CI, 1.24, 8.43. *P* = 0.017).

The predictive performance of the HE thresholds for basal ganglia ICH is shown in Table 4. All HE thresholds showed higher specificity than sensitivity, and the two absolute growth thresholds showed a high accuracy rate of 70.16%. Hematoma growth > 6 ml had the highest specificity and positive predictive value. The predictive values of relative growth > 33% were lower compared to the absolute growth thresholds except for the specificity. Although hematoma growth > 3 ml or >33% showed the highest sensitivity and negative predictive value, the accuracy of their combination was not better than that of the absolute hematoma growth thresholds.

As shown in Figure 3, the correlations between most variables were similar in thalamic and basal ganglia ICH. However, PLIC involvement and HE (growth > 3 ml or >33%) had a higher correlation in thalamic ICH compared to basal ganglia ICH (0.24 vs. 0.03). Thus, the correlation between PLIC involvement and mRS > 3 and between HE and mRS > 3 varied at the two ICH locations. In addition, thalamic ICH without PLIC involvement also had a lower possibility of HE (*P* = 0.009). No such difference was seen in basal ganglia ICH (Table 5).

## 4. Discussion

This retrospective study demonstrated the differential prognostic impact of HE in patients with deep ICH. Thalamic ICH had a smaller volume at baseline CT and a low risk of HE but was more likely to initially involve PLIC (Figure 4). We further found that in the absence of PLIC involvement, thalamic ICH was less likely to develop HE. Since baseline hemorrhage volume and PLIC involvement both correlate significantly with mRS > 3 [20], in multivariate analysis, the effect of HE on functional prognosis was largely replaced by the two variables; the adjusted ORs of thalamic hematoma growth were not significant, whereas basal ganglia ICH had a lower incidence of PLIC involvement at both baseline and follow-up CT and tended to absolute growth leading to an increase in hematoma volume. So, all HE thresholds were independent risk factors for the poor functional outcome in basal ganglia ICH, and absolute ICH growth thresholds showed greater predictive power.

Consistent with previous studies [11, 21], advanced age, GCS score, presence of IVH, and PLIC involvement were also associated with mRS > 3. In our study, 95.95% (403/420) of the patients were found with hypertension. Though patients with poor outcome had higher systolic BP on admission, the difference was not significant. Recent evidence [22, 23] suggested that intensive BP reduction (systolic BP < 140 mmHg), especially within ultraearly time frame, could attenuate HE and improve outcome in ICH patients, whereas the treatment in this study was to reduce and maintain a systolic BP target of 160 mmHg.

The incidence of HE was lower in thalamic versus basal ganglia ICH, although the difference was not significant when using the relative growth threshold > 33%. Previous studies [24, 25] have associated HE with large hematomas. The lower volume of thalamic ICH (9.55 ± 6.85 ml) compared to that of basal ganglia ICH may be attributed to the lower incidence of HE.

Early identification of different HE thresholds might be helpful to adopt different strategies for ICH patients at high risk of hematoma growth. An ideal definition of HE in trials of hemostatic therapies should perform well in capturing a reasonable proportion of patients and must exceed MDD [17]. ICH absolute growth of 6 ml and relative growth of 33% have been frequently used as the minimally important threshold of HE to avoid measurement errors [11, 18, 24]. However, Rodriguez-Luna et al. calculated hematoma volume using computerized planimetry software and found that the MDDs ranged from 0.56 ml to 2.52 ml in the intra- and interobserver tests, respectively, when the hemorrhage volumes were less than 30 ml [26]. A recent study found that patients with deep ICH was vulnerable to the deleterious effects of small threshold of HE [27]. In our study, baseline volume of deep ICH was 17.94 ± 13.91 ml, and we used the similar method to measure hematoma volume and found that the threshold of ICH volume > 3 ml was a reliable index.

For predicting mRS > 3 in patients with basal ganglia ICH, the absolute hematoma growth thresholds were more accurately predictive compared to the relative threshold, although their combination was not superior. The positive predictive value increased at the expense of sensitivity, which may exclude some patients who developed HE. The ICH volume in the follow-up CT had increased by 3.68 ml and 3.41 ml in two patients (designated A and B, respectively, in Figure 5), even though the relative increase in hematoma volume was only 24.22% in patient B, and the mRS of patient B rose to 4 after HE. We also observed that thalamic ICH without PLIC involvement was less likely to develop HE, which can be attributed to the lower pressure of the medial thalamic artery rupture that results in smaller ICH volume and a lower incidence of HE than that in the lateral thalamus. In addition, the inherent structural differences between the medial and lateral thalamus may also limit HE. As opposed to dense gray matter containing cell nuclei, thalamic ICH involving PLIC is likely to expand toward the loose white matte.

Our study specifically assessed the relationship between HE and functional outcome separately among thalamic ICH and basal ganglia ICH groups, making it more of a “location-specific” evaluation method, rather than using a “one size fits all” method for all HE. Several limitations of the study ought to be addressed. Some potential covariates were not recorded or incomplete, such as the National Institutes of Health Stroke Scale (NIHSS) scores. INR and platelet count were missed in nearly half of the patients, but the remaining patients all had medical records with normal coagulation function. Furthermore, the time from symptom onset to baseline CT (median, 3 hours; IQR, 2-4 hours) in our study was longer than that in other studies [3, 17], which also affects the frequency of HE [28]. In addition, we excluded patients without follow-up imaging, which may have biased the effect of ICH location on the early clinical outcome. The patients that underwent hematoma stereotactic evacuation or additional craniectomy had a higher survival rate compared to patients who received conservative treatment [12], which may have partially affected the results. The primary outcome of this study was the mRS at the short follow-up of 30 days, which is a measure of motor disability and neglects quality of life. Finally, we did not consider IVH expansion that is strongly predictive of poor outcome [29, 30]. Therefore, the overall and long-term prognoses of these patients need to be studied further to validate our findings.

In conclusion, HE has different prognostic impact in thalamic and basal ganglia ICH. HE is not an independent risk factor for the poor functional outcome in thalamic ICH but robustly predicts a poor outcome in basal ganglia ICH regardless of growth threshold, and absolute growth is more predictive of short-term poor functional outcome than relative growth.

## Figures and Tables

**Figure 1:** Flowchart showing inclusion and exclusion criteria.

**Figure 2:** Receiver operating characteristic (ROC) curves for absolute growth and relative growth.

**Figure 3:** Correlation coefficient matrix of the covariates and poor outcomes: (a) thalamic ICH and (b) basal ganglia ICH. GCS: Glasgow Coma Scale; BV: baseline volume; PLICI: posterior limb of internal capsule involvement; IVH: intraventricular hemorrhage; HE: hematoma expansion (growth > 3 ml or >33%).

**Figure 4:** Thalamic hemorrhage with the posterior limb of internal capsule involvement. Patient A is a 71-year-old male with right thalamic hemorrhage, the baseline CT (A1) scan was performed 1.5 hours after symptom onset, and the follow-up CT (A2) showed that hemorrhage had not expanded. Patient B is a 55-year-old woman with right thalamic hemorrhage, and the follow-up CT (B2) showed hemorrhage increased by 3.66 ml than the initial volume (B1).

**Figure 5:** Basal ganglia hemorrhage. Patient A is a 59-year male with left basal ganglia hemorrhage, the baseline CT (A1) scan was performed 40 minutes after symptom onset and 24 hours later, the hemorrhage increased by 3.68 ml (A2), and the mRS was 2 at day 30. Patient B is a 54-year male, the baseline CT (A1) scan was performed 2 hours after symptom onset, and hemorrhage volume was 14.08 ml; the follow-up CT (B2) showed that hemorrhage increased by 3.41 ml (24.22%), and mRS was 4 at day 30.

**Table 1:** Baseline characteristics of the ICH locations.

Characteristics	Thalamic ICH (*N* = 147)	Basal ganglia ICH (*N* = 273)	*P* value
Age (years)	64 (55-75)	59 (50-67)	<0.001
Male, *N* (%)	88 (59.86%)	187 (68.50%)	0.076
Risk factor			
Diabetes, *N* (%)	15 (10.20%)	25 (9.16%)	0.727
Antiplatelet medications, *N* (%)	6 (4.08%)	11 (4.03%)	0.997
Current smoking, *N* (%)	13 (8.84%)	26 (9.52%)	0.783
Daily alcohol drinking, *N* (%)	5 (3.4%)	20 (7.35%)	0.097
Clinical information			
GCS score	12 (8-14)	12 (9-14)	0.551
Systolic BP (mmHg)	177.94 ± 26.16	178.23 ± 28.42	0.917
Diastolic BP (mmHg)	100.27 ± 17.66	102.86 ± 18.28	0.162
Symptom onset to baseline CT (hour)	3 (2-4)	3 (2-4)	0.667
Laboratory testing			
Platelet count (10^9^/L)^a^	202.83 ± 71.99	206.99 ± 73.3	0.458
International normalized ratio^b^	1.04 ± 0.12	1.04 ± 0.12	0.431
CT findings on baseline CT			
ICH volume (ml)	9.55 ± 6.85	17.95 ± 13.92	<0.001
PLIC involvement, *N* (%)	85 (57.82%)	55 (20.15%)	<0.001
Presence of IVH, *N* (%)	108 (73.47%)	61 (22.34%)	<0.001
CT findings on follow-up CT			
ICH volume (ml)	12.92 ± 15.37	24.79 ± 22.56	<0.001
PLIC involvement, *N* (%)	88	71	<0.001
Presence of IVH, *N* (%)	108	79	<0.001
HE			
Growth > 6 ml, *N* (%)	21 (14.29%)	80 (29.30%)	0.001
Growth > 33%, *N* (%)	31 (21.09%)	80 (29.41%)	0.065
Treatment^c^			
External ventricular drainage, *N* (%)	23 (16.31%)	15 (5.81%)	0.001
ICH stereotactic evacuation or craniectomy, *N* (%)	6 (4.26%)	46 (17.83%)	<0.001
Outcome^c^			
mRS > 3, *N* (%)	84 (59.57%)	129 (50.0%)	0.067
Mortality, *N* (%)	12 (8.51%)	33 (12.79%)	0.196

Abbreviations: BP: blood pressure; CT: computed tomography; HE: hematoma expansion; mRS: modified Rankin scale; ICH: intracerebral hemorrhage; PLIC: posterior limb of internal capsule; IVH: intraventricular hemorrhage; GCS: Glasgow Coma Scale. Normally distributed continuous variables are summarized by means ± SD, and skewed continuous variables are presented as medians and interquartile ranges (IQR). ^a^Missing 213 patients. ^b^Missing 206 patients. ^c^21 patients lost to follow-up.

**Table 2:** Logistic regression analysis with poor functional outcome as a dependent variable in thalamic ICH (*N* = 141).

	mRS ≤ 3 (*n* = 57, 40.43%)	mRS > 3 (*n* = 84, 59.57%)	Univariate analysis	*P* value	Multivariable analysis	*P* value
			OR (95% CI)		OR (95% CI)	
Age (year)	62 (54-70)	67 (59-77)	1.03 (1.01, 1.06)^∗^	0.018	1.06 (1.02, 1.12)^∗^	0.01
Male, *N* (%)	38 (66.67%)	45 (53.57%)	0.57 (0.28, 1.15)	0.121	—	—
GCS score	13 (12-14)	10 (7-12)	0.72 (0.62, 0.83)^∗^	<0.001	0.78 (0.64, 0.95)^∗^	0.016
History of diabetes, *N* (%)	4 (7.02%)	11 (13.10%)	2.0 (0.64, 7.52)	0.258	—	—
Current smoking, *N* (%)	5 (8.77%)	8 (9.52%)	1.09 (0.35, 3.80)	0.880	—	—
Daily alcohol drinking, *N* (%)	1 (1.75%)	4 (4.76%)	2.80 (0.40, 55.56)	0.363	—	—
Antiplatelet medications, *N* (%)	2 (3.51%)	4 (4.76%)	1.38 (0.26, 10.16)	0.719	—	—
Systolic BP (mmHg)	172.49 ± 25.11	181.14 ± 25.99	1.01 (1.00, 1.03)	0.054	1.02 (0.99, 1.04)	0.126
Diastolic BP (mmHg)	100.84 ± 20.27	99.38 ± 15.01	1.0 (0.98, 1.01)	0.622	—	—
Symptom onset to baseline CT (hour)	3 (2-4)	3 (2-4)	0.96 (0.78, 1.18)	0.686	—	—
Baseline ICH volume (ml)	5.70 ± 2.87	11.79 ± 6.59	1.38 (1.23, 1.59)^∗^	<0.001	1.26 (1.08, 1.51)^∗^	0.006
PLIC involvement, *N* (%)	11 (19.3%)	66 (78.57%)	15.33 (6.85, 37.01)^∗^	<0.001	11.69 (4.05, 38.27)^∗^	<0.001
Intraventricular hemorrhage, *N* (%)	32 (56.14%)	70 (83.33%)	3.91 (1.82, 8.68)^∗^	<0.001	1.62 (0.52, 4.89)	0.383
Hematoma growth^#^ > 3 ml, *N* (%)	4 (7.02%)	21 (25.0%)	4.42 (1.56, 15.85)^∗^	<0.001	1.36 (0.28, 7.92)	0.715
Hematoma growth^#^ > 6 ml, *N* (%)	2 (3.51%)	17 (20.24%)	6.98 (1.89, 45.22)^∗^	0.012	1.44 (0.22, 13.18)	0.167
Hematoma growth^#^ > 33%, *N* (%)	6 (10.53%)	21 (25.0%)	2.83 (1.12, 8.19)^∗^	0.037	1.66 (0.37, 8.21)	0.512

Abbreviations: OR: odds ratio; CI: confidence interval; ICH: intracerebral hemorrhage; BP: blood pressure; PLIC: posterior limb of internal capsule; GCS: Glasgow Coma Scale. ^#^The independent variables were brought into multivariable logistic regression, respectively. ^∗^Statistically significant finding. Normally distributed continuous variables are summarized by means ± SD, and skewed continuous variables are presented as medians and interquartile ranges (IQR).

**Table 3:** Logistic regression analysis with poor functional outcome as a dependent variable in basal ganglia ICH (*N* = 258).

	mRS ≤ 3 (*n* = 129, 50%)	mRS > 3 (*n* = 129, 50%)	Univariate analysis	*P* value	Multivariable analysis	*P* value
			OR (95% CI)		OR (95% CI)	
Age (year)	55 (48-65)	60 (52-70)	1.04 (1.03, 1.06)^∗^	<0.001	1.06 (1.03, 1.10)^∗^	<0.001
Male, *N* (%)	92 (71.32%)	84 (65.12%)	0.75 (0.44, 1.27)	0.285	—	—
GCS score	13 (10-14)	10 (7-12)	0.71 (0.63, 0.78)^∗^	<0.001	0.78 (0.67, 0.89)^∗^	<0.001
History of diabetes, *N* (%)	9 (6.98%)	14 (10.85%)	1.62 (0.69, 3.81)	0.275	—	—
Current smoking, *N* (%)	11 (8.53%)	14 (10.85%)	1.31 (0.58, 2.94)	0.528	—	—
Daily alcohol drinking, *N* (%)	10 (7.75%)	8 (6.20%)	0.79 (0.31, 2.01)	0.625	—	—
Antiplatelet medications, *N* (%)	2 (1.55%)	7 (5.43%)	3.64 (0.82, 16.27)	0.086	0.93 (0.11, 10.37)	0.861
Systolic BP (mmHg)	176.99 ± 27.78	181.33 ± 28.60	1.02 (1.0, 1.04)	0.075	1.0 (0.98, 1.01)	0.614
Diastolic BP (mmHg)	103.75 ± 16.20	102.68 ± 19.27	1.01 (0.98, 1.04)	0.581	—	—
Symptom onset to baseline CT (hour)	3 (2-4)	3 (2-4)	0.87 (0.64, 1.18)	0.387	—	—
Baseline ICH volume (ml)	11.49 ± 8.44	24.51 ± 15.61	1.15 (1.07, 1.26)^∗^	<0.001	1.10 (10.6, 1.14)^∗^	<0.001
PLIC involvement, *N* (%)	11 (8.35%)	42 (32.56%)	5.18 (2.55, 10.51)^∗^	<0.001	7.56 (2.82, 22.2)^∗^	<0.001
Intraventricular hemorrhage, *N* (%)	14 (10.85%)	45 (34.88%)	4.40 (2.28, 8.47)^∗^	<0.001	3.16 (1.24, 8.43)^∗^	0.017
Hematoma growth^#^ > 3 ml, *N* (%)	24 (18.60%)	76 (58.91%)	6.27 (3.57, 10.01)^∗^	<0.001	7.56 (3.5, 17.34)^∗^	<0.001
Hematoma growth^#^ > 6 ml, *N* (%)	13 (10.08%)	65 (50.39%)	9.06 (4.67, 17.55)^∗^	<0.001	8.09 (3.48, 20.26)^∗^	<0.001
Hematoma growth^#^ > 33%, *N* (%)	19 (14.73%)	58 (44.96)	4.72 (2.64, 8.77)^∗^	<0.001	10.68 (4.54, 27.33)^∗^	<0.001

Abbreviations: OR: odds ratio; CI: confidence interval; ICH: intracerebral hemorrhage; BP: blood pressure; PLIC: posterior limb of internal capsule; GCS: Glasgow Coma Scale. ^#^The independent variables were brought into multivariable logistic regression, respectively. ^∗^Statistically significant finding. Normally distributed continuous variables are summarized by means ± SD, and skewed continuous variables are presented as medians and interquartile ranges (IQR).

**Table 4:** Performance of the HE thresholds for the prediction of the poor outcome (mRS > 3)^a^ in basal ganglia ICH.

HE	Frequency, *N* (%)	Sensitivity (%)	Specificity (%)	PPV (%)	NPV (%)	Accuracy (%)
Growth > 3 ml	100 (38.76)	58.91	81.4	76	66.46	70.16
Growth > 6 ml	78 (30.23)	50.39	89.92	83.33	64.44	70.16
Growth > 33%	77 (29.84)	44.96	85.27	75.32	60.77	65.12
Growth > 3 ml or 33%	105 (40.7)	60.47	79.07	74.29	66.67	69.76
Growth > 6 ml or 33%	90 (34.88)	54.26	84.5	77.78	64.88	69.38

Abbreviation: mRS = modified Rankin scale; HE = hematoma expansion; PPV = positive predictive value; NPV = negative predictive value. ^a^*N* = 258.

**Table 5:** The relationship of hematoma expansion with the posterior limb of internal capsule involvement in deep ICH.

HE (growth > 3 ml or >33%)	Posterior limb of internal capsule involvement, *N* (%)					
	Thalamic ICH (*N* = 147)			Basal ganglia ICH (*N* = 273)		
	Yes	No	*P*	Yes	No	*P*
Yes	25 (17.0%)	7 (4.76%)	0.009	23 (8.43%)	86 (31.50%)	0.749
No	60 (40.82%)	55 (37.42%)		32 (11.72%)	132 (48.35%)	

Abbreviations: ICH: intracerebral hemorrhage; HE: hematoma expansion.

## Data Availability

The datasets used and analyzed during the current study are available from our corresponding author on reasonable request.

## References

[1] Neisewander B. L., Hu K., Tan Z. (2018). Location of thalamic hemorrhage impacts prognosis. *World Neurosurgery*.

[2] Li Q., Liu Q.-J., Yang W.-S. (2017). Island sign: an imaging predictor for early hematoma expansion and poor outcome in patients with intracerebral hemorrhage. *Stroke*.

[3] Li Q., Shen Y. Q., Xie X. F. (2019). Expansion-prone hematoma: defining a population at high risk of hematoma growth and poor outcome. *Neurocritical Care*.

[4] Xie H., Ma S., Wang X., Zhang X. (2020). Noncontrast computer tomography–based radiomics model for predicting intracerebral hemorrhage expansion: preliminary findings and comparison with conventional radiological model. *European Radiology*.

[5] Ma C., Zhang Y., Niyazi T. (2019). Radiomics for predicting hematoma expansion in patients with hypertensive intraparenchymal hematomas. *European Journal of Radiology.*.

[6] Orito K., Hirohata M., Nakamura Y. (2016). Leakage sign for primary intracerebral hemorrhage: a novel predictor of hematoma growth. *Stroke*.

[7] He Q., Zhou Y., Wang F., Li B., Cheng Y., Xie Z. Y. (2019). Blood type O predicts hematoma expansion in patients with intracerebral hemorrhage. *Journal of stroke and cerebrovascular diseases*.

[8] Eslami V., Tahsili-Fahadan P., Rivera-Lara L. (2019). Influence of intracerebral hemorrhage location on outcomes in patients with severe intraventricular hemorrhage. *Stroke*.

[9] Delcourt C., Sato S., Zhang S. (2017). Intracerebral hemorrhage location and outcome among INTERACT2 participants. *Neurology*.

[10] Sreekrishnan A., Dearborn J. L., Greer D. M. (2016). Intracerebral hemorrhage location and functional outcomes of patients: a systematic literature review and meta-analysis. *Neurocritical Care*.

[11] Yogendrakumar V., Demchuk A. M., Aviv R. I. (2017). Location of intracerebral haemorrhage predicts haematoma expansion. *European Stroke Journal*.

[12] Safatli D. A., Gunther A., Schlattmann P., Schwarz F., Kalff R., Ewald C. (2016). Predictors of 30-day mortality in patients with spontaneous primary intracerebral hemorrhage. *Surgical Neurology International*.

[13] Löppönen P., Qian C., Tetri S., Juvela S. (2014). Predictive value of C-reactive protein for the outcome after primary intracerebral hemorrhage. *Journal of Neurosurgery*.

[14] Roh D., Sun C. H., Schmidt J. M. (2018). Primary intracerebral hemorrhage: a closer look at hypertension and cerebral amyloid angiopathy. *Neurocritical Care*.

[15] Nakagawa K., King S. L., Seto T. B. (2018). Optimal hematoma volume cut points to predict functional outcome after basal ganglia and thalamic hemorrhages. *Frontiers in Neurology*.

[16] Jafari M., di Napoli M., Lattanzi S. (2019). Serum magnesium level and hematoma expansion in patients with intracerebral hemorrhage. *Journal of the Neurological Sciences*.

[17] Dowlatshahi D., Demchuk A., Flaherty M., Ali M., Lyden P., Smith E. J. N. (2011). Defining hematoma expansion in intracerebral hemorrhage: relationship with patient outcomes. *Neurology*.

[18] Roh D., Sun C.-H., Murthy S. (2019). Hematoma expansion differences in lobar and deep primary intracerebral hemorrhage. *Neurocritical Care*.

[19] Perkins N. J., Schisterman E. F. (2006). The inconsistency of "optimal" cutpoints obtained using two criteria based on the receiver operating characteristic curve. *American journal of epidemiology.*.

[20] Czernicki T., Maj E., Podgórska A. (2017). Diffusion tensor tractography of pyramidal tracts in patients with brainstem and intramedullary spinal cord tumors: relationship with motor deficits and intraoperative MEP changes. *Journal of Magnetic Resonance Imaging*.

[21] Ironside N., Chen C. J., Dreyer V., Christophe B., Buell T. J., Connolly E. S. (2020). Location-specific differences in hematoma volume predict outcomes in patients with spontaneous intracerebral hemorrhage. *International Journal of Stroke*.

[22] Li Q., Warren A. D., Qureshi A. I. (2020). Ultra-early blood pressure reduction attenuates hematoma growth and improves outcome in intracerebral hemorrhage. *Annals of Neurology*.

[23] Morotti A., Boulouis G., Romero J. M. (2017). Blood pressure reduction and noncontrast CT markers of intracerebral hemorrhage expansion. *Neurology*.

[24] Dowlatshahi D., Smith E. E., Flaherty M. L. (2011). Small intracerebral haemorrhages are associated with less haematoma expansion and better outcomes. *International Journal of Stroke*.

[25] Barras C. D., Tress B. M., Christensen S. (2009). Density and shape as CT predictors of intracerebral hemorrhage growth. *Stroke*.

[26] Rodriguez-Luna D., Boyko M., Subramaniam S. (2016). Magnitude of hematoma volume measurement error in intracerebral hemorrhage. *Stroke*.

[27] Roh D., Boehme A., Young C. (2020). Hematoma expansion is more frequent in deep than lobar intracerebral hemorrhage. *Neurology*.

[28] al-Shahi Salman R., Frantzias J., Lee R. J. (2018). Absolute risk and predictors of the growth of acute spontaneous intracerebral haemorrhage: a systematic review and meta-analysis of individual patient data. *The Lancet Neurology*.

[29] Yogendrakumar V., Ramsay T., Fergusson D. A. (2020). Redefining hematoma expansion with the inclusion of intraventricular hemorrhage growth. *Stroke*.

[30] Yogendrakumar V., Ramsay T., Fergusson D. (2019). New and expanding ventricular hemorrhage predicts poor outcome in acute intracerebral hemorrhage. *Neurology*.

